The article "Long noncoding RNA HOXA-AS2 promotes non-small cell lung cancer progression by regulating miR-520a-3p" was retracted in 2022. Reasons: duplicated images; signs of a paper mill.

# Long noncoding RNA HOXA-AS2 promotes non-small cell lung cancer progression by regulating miR-520a-3p

**DOI:** 10.1042/BSR20190283

**Published:** 2019-05-31

**Authors:** Yunpeng Liu, Xingyu Lin, Shiyao Zhou, Peng Zhang, Guoguang Shao, Zhiguang Yang

**Affiliations:** 1 Department of Thoracic Surgery, The First Hospital of Jilin University, Changchun, Jilin 130021, P.R. China; 2 Department of Anaesthesia, The First Hospital of Jilin University, Changchun, Jilin 130021, P.R. China

**Keywords:** HOXA-AS2, Long non-coding RNA, miR-520a-3p, non-small cell lung cancer, proliferation

## Abstract

***Background:*** The HOXA cluster antisense RNA 2 (HOXA-AS2) has recently been discovered to be involved in carcinogenesis in multiple cancers. However, the role and underlying mechanism of HOXA-AS2 in non-small cell lung cancer (NSCLC) yet need to be unraveled. ***Methods:*** HOXA-AS2 expression in NSCLC tissues and cell lines was detected using quantitative real-time PCR (qRT-PCR). Furthermore, the effects of HOXA-AS2 on NSCLC cell proliferation, apoptosis, migration, and invasion were assessed by MTS, flow cytometry, wound healing and transwell invasion assays, respectively. Starbase2.0 predicted and luciferase reporter and RNA immunoprecipitation (RIP) assays were used to validate the association of HOXA-AS2 and miR-520a-3p in NSCLC cells. ***Results:*** Our results revealed that HOXA-AS2 in NSCLC tissues were up-regulated and cell lines, and were associated with poor prognosis and overall survival. Further functional assays demonstrated that HOXA-AS2 knockdown significantly inhibited NSCLC cell proliferation, induced cell apoptosis and suppressed migration and invasion. Starbase2.0 predicted that HOXA-AS2 sponge miR-520a-3p at 3′-UTR, which was confirmed using luciferase reporter and RIP assays. miR-520a-3p expression was inversely correlated with HOXA-AS2 expression in NSCLC tissues. In addition, miR-520a-3p inhibitor attenuated the inhibitory effect of HOXD-AS2-depletion on cell proliferation, migration and invasion of NSCLC cells. Moreover, HOXA-AS2 could regulate HOXD8 and MAP3K2 expression, two known targets of miR-520a-3p in NSCLC. ***Conclusion:*** These findings implied that HOXA-AS2 promoted NSCLC progression by regulating miR-520a-3p, suggesting that HOXA-AS2 could serve as a therapeutic target for NSCLC.

## Introduction

Non-small cell lung cancer (NSCLC), accounting for approximately 80% of lung cancers, is one of the most malignant tumors worldwide with a low overall 5-year survival rate [1,2]. Although great progress has been made in the study of the NSCLC, the molecular mechanism in the occurrence and progression of NSCLC still remains elusive [3]. Thus, there is an urgent need to explore molecular mechanism of pathogenesis and progression of NSCLC to find novel targets for effective therapies.

Long noncoding RNAs (lncRNAs) with length more than 200 nucleotides are a type of noncoding RNAs without protein-encoding ability [4]. LncRNAs have been reported to be involved in multiple cellular processes, such as cell proliferation, apoptosis, cycle and invasion [5,6]. Growing evidence demonstrated that the aberrant expression of lncRNAs were associated with tumorigenesis and development of various types of cancer, and functioned as either oncogenes or tumor suppressors [7,8]. Number of cancer-related lncRNAs was identified to play crucial roles in initiation and development of NSCLC, indicating that lncRNAs could serve as diagnostic marker and therapy target for NSCLC [9,10].

HOXA cluster antisense RNA 2 (HOXA-AS2), a discovered lncRNA located between the HOXA3 and HOXA4 genes in the HOXA cluster [11], has been reported to be involved in regulation of endothelium inflammation and formation of osteogenesis [12,13]. A body of evidence suggested that HOXA-AS2 expression was up-regulated in hepatocellular carcinoma [14], bladder cancer [15], papillary thyroid cancer [16], osteosarcoma [17], pancreatic cancer [18], colorectal cancer [19], breast cancer [20] and gastric cancer [21], suggesting that it played tumor-promoting role in these cancers. However, little is known about the expression status, biological function and underlying mechanism on NSCLC carcinogenesis or metastasis.

The aims of the current study, therefore, were to explore the role of HOXA-AS2 in the regulation of proliferation, apoptosis, migration and invasion of NSCLC and investigate the association between HOXA-AS2 and its target miRNAs to uncover the underlying regulatory mechanisms of NSCLC development.

## Materials and methods

### Tissue collection

Fifty-two pairs of NSCLC tissues and corresponding adjacent normal tissues were harvested from patients who were diagnosed with NSCLC and underwent surgery in Department of Thoracic Surgery, The First Hospital of Jilin University (Changchun, China). None of the patients received local or systemic therapy prior to surgery. All tissues were histologically confirmed by our hospital, and stored in liquid nitrogen until use. Clinicopathologic characteristics of these patients were listed in Table 1. This research was conducted as per the Declaration of Helsinki, after acceptance from the Research Ethics Committee of Jilin University. Written informed consent was signed by all patients.

**Table 1:** Correlation between clinicopathological features and HOXA-AS2 expression in NSCLC

Variables	Number of cases	HOXA-AS2 expression		*P*-value
		Low	High	
Age (years)				*P*=0.7852
<60	22	10	12	
≥60	30	15	15	
Gender				*P*=0.7804
Male	29	13	16	
Female	23	12	11	
TNM stage				*P*=0.0001
T1–T2	37	24	13	
T3–T4	15	1	14	
Tumor size				*P*=0.5737
<3 cm	33	17	16	
≥3 cm	19	8	11	
Lymph node metastasis				*P*=0.0008
No	36	23	13	
Yes	16	2	14	

Abbreviation: TNM, tumor-node metastasis.

### Cell culture and transfection

Four human NSCLC cell lines (SPC-A1, NCI-H358, A549 and PC9) and normal lung 16HBE epithelial cells were purchased from Shanghai Institutes for Biological Sciences, China. All cells were grown in DMEM (HyClone, Logan, UT, U.S.A.) supplemented with 10% fetal bovine serum (FBS; Gibco, NY, U.S.A.), 100 U/ml penicillin and 100 mg/ml streptomycin (Sigma, U.S.A.) in a humidified atmosphere containing 5% CO_2_ at 37°C in incubator (Memmert, Germany).

Three small interfering RNAs (siRNAs) against HOXA-AS2 (si-HOXA-AS2#1, si-HOXA-AS2#2 and si-HOXA-AS2#3) and non-target siRNA control (si-NC) were designed and synthesized from GenePharma (Shanghai, China). The miR-520a-3p mimic, negative control mimic (miR-NC), miR-520a-3p inhibitor (miR-520a-3p in) were bought from Ribobio (Guangzhou, China). A549 cells were transfected by the above-mentioned siRNA, mimic and inhibitor using Lipofectamine 2000 (Life Technologies) as per the manufacturer’s instructions.

### RNA isolation and quantitative real-time PCR

Total RNA was extracted from cultured cells and NSCLC tissues or adjacent normal tissues using TRIzol reagent (Thermo Fisher Scientific, Carlsbad, CA, U.S.A.). RNA samples were reverse transcribed into complementary DNA (cDNA) using TaqMan MicroRNA Reverse Transcription kit (Thermo Fisher Scientific) or PrimeScript™ RT Master Mix (Takara, Dalian, China), then quantitated using TaqMan microRNA assays kits (Thermo Fisher Scientific) or FastStart Universal SYBR-Green Master Mix (Roche, Basel, Switzerland) on a 7900HTfast Real-time PCR system (Applied Biosystems, Foster City, CA). The primers used in the present study are listed in Table 2. The relative expression levels were calculated using 2^−ΔΔ*C*^_t_ method following normalization against U6 for miR-520a-3p or GAPDH for *HOXA-AS2, HOXD8* and *MAP3K2* mRNAs.

**Table 2:** Real-time PCR primers used for mRNA expression analysis

Target gene	Primers (5′–3′)
*U6*	F- TCCGATCGTGAAGCGTTC
	R- GTGCAGGGTCCGAGGT
*miR-520a-3p*	F- GCCACCACCATCAGCCATAC
	R- GCACATTACTCTACTCAGAAGGG
*HOXA-AS2*	F- GAAAACCACGCTTTTCCCGT
	R- CCTTTAGGCCTTCGCAGACA
*HOXD8*	F- CCTGACTGTAAATCGTCCAGTGGTA
	R- AGTTTGGAAGCGACTGTAGGTTTG
*MAP3K2*	F- CCCCAGGTTACATTCCAGATGA
	R- GCATTCGTGATTTTGGATAGCTC
*GAPDH*	F- AAGGTGAAGGTCGGAGTCAA
	R- AATGAAGGGGTCATTGATGG

Abbreviations: F, forward; mRNA, messenger RNA; PCR, polymerase chain reaction; R, reverse.

### Cell proliferation assay

Transfected cells (5 × 10^3^ per well in 100 μl) were seeded into 96-well plates cultured for 24–72 h. In specific times (24, 48 and 72 h), cell proliferation was examined using CellTiter 96®AQueous One Solution Cell Proliferation Assay kit (MTS; Promega, Madison, WI, U.S.A.) following the manufacturer’s instructions. The absorbance at 490 nm was detected using a Benchmark Plus microplate spectrometer (Bio-Rad Laboratories, Hercules, CA, U.S.A.).

### Cell apoptosis assay

Cells were collected using trypsinization at 48 h post-transfection. Then cells were stained with FITC-Annexin V and Propidium iodide (PI) using an Annexin-V-FITC apoptosis detection kit (BD Bioscience, Franklin Lakes, NJ, U.S.A.). Data were acquired using an FACSCalibur flow cytometry (BD Biosciences). The apoptosis ratio was analyzed with CellQuest 3.0 software (BD Biosciences).

### Wound healing assay

To determine the effect of HOXA-AS2 on cell migration, wound healing assay was conducted. Briefly, transfected cells were seeded in 12-well plates and grown to 80–90% confluence. Then, identical wound was created using a sterile 10-μl pipette tip. To remove detached cells, cells were washed with PBS solution, following culturing in a serum-free medium for 24 h. Images were taken at 0 and 24 h after wounding using a light microscope (Olympus Corp., Tokyo, Japan).

### Transwell invasion assay

Cell invasion abilities were determined using Boyden chamber invasion assay (24-well plate format). In brief, the transfected cells (5 × 10^4^ cells each well) were plated in upper well of Corning Costar Transwell 24-well plates (8-μm pores; Corning, U.S.A.) pre-coated with Matrigel (BD, Biosciences) and cultured in serum-free medium. DMEM with 20% FBS was placed in the bottom wells as a chemoattractant. After 48 h of incubation at 37°C, a cotton swab was used to remove the noninvasive cells remaining on upper well, while invaded cells were fixed and stained in 0.1% Crystal Violet for 5 min. The stained cells were captured using a light microscope (Nikon) and counted in five randomly selected fields by software Image Pro Plus 6.0.

### Luciferase reporter assay

The sequence fragment of HOXA-AS2 (WT-HOXA-AS2) containing the putative target sites for miR-520a-3p were synthesized and inserted into the pmirGLO vector (Promega Corp., Madison, WI, U.S.A.). The mutant miR-520a-3p binding sites for HOXA-AS2 (MT-HOXA-AS2) were generated using QuikChange II Site-Directed Mutagenesis Kit (Stratagene, La Jolla, CA, U.S.A.). For luciferase reporter assay, A549 cells were co-transfected with reporter vector containing WT-HOXA-AS2 or MT-HOXA-AS2 and miR-520a-3p mimic or miR-NC. At 48 h after transfection, Dual-Luciferase reporter assay system (Promega) was used to detect the activities of *Renilla* luciferase and firefly luciferase. The relative luciferase activity was standardized to *Renilla* luciferase activity.

### RNA immunoprecipitation assay

To investigate if HOXA-AS2 and miR-520a-3p were associated with the RNA-induced silencing complex (RISC), RNA immunoprecipitation (RIP) experiment was conducted using the Magna RIP Kit (Millipore, Billerica, MA, U.S.A.) with the Ago2 antibody (Abcam, U.S.A.) according to the manufacturer’s protocol. Normal mouse IgG (Abcam) used in the present study served as a control. The expression levels of HOXA-AS2 and miR-520a-3p in the precipitates were measured by quantitative real-time PCR (qRT-PCR) as mentioned above.

### Statistical analysis

Quantitative data are expressed as the mean ± standard deviation (S.D.) from at least three independent repeats of the experiments, and were analyzed using SPSS v. 19.0 (IBM Corp., Armonk, NY, U.S.A.). Student’s *t*test was used to assess significant differences between two groups. One-way analysis of variance was employed to estimate the significant differences among multiple groups. The correlation in a dataset was analyzed using Spearman’s correlation analysis. Kaplan–Meier method and the log-rank test were used to determine overall survival ratio. A *P*-value less than 0.05 was considered as statistically significant.

## Results

### HOXA-AS2 was up-regulated and associated with poor prognosis of patients with NSCLC

To investigate the expression status of HOXA-AS2 in NSCLC, we detected the expression of HOXA-AS2 in NSCLC tissues and adjacent normal tissues from 52 patients with NSCLC. The results of qRT-PCR revealed that the expression of HOXA-AS2 were up-regulated in NSCLC tissues compared with adjacent normal tissues (Figure 1A). In consistence, HOXA-AS2 expression was also elevated in four NSCLC cell lines (SPC-A1, NCI-H358, A549 and PC9) relative to normal lung 16HBE epithelial cells (Figure 1B). Additionally, our results demonstrated that HOXA-AS2 mainly existed in the cytoplasm of NSCLC cells (Figure 1C). To investigate the association with HOXA-AS2 and patient’s clinical features, we divided these NSCLC tissues into two groups: High expression of HOXA-AS2 (*n*=27) and Low expression of HOXA-AS2 groups (*n*=25) based on median level of HOXA-AS2. We found that increased HOXA-AS2 was closely associated with tumor-node metastasis (TNM) stage and lymph node metastasis (Table 1). However, no correlation was observed in patient’s age, gender and tumor size (Table 1). In addition, we found patients with high expression of HOXA-AS2 displayed poor overall survival rate (Figure 1D), suggesting HOXA-AS2 might be a prognostic indicator. These results suggested that HOXA-AS2 might play a key role in NSCLC development.

**Figure 1:** HOXA-AS2 was up-regulated and associated with poor prognosis of patients with NSCLC (**A**) The expression of HOXA-AS2 in 52 pairs of NSCLC tissues and adjacent normal tissues were examined by qRT-PCR. (**B**) The expression of HOXA-AS2 were measured in four NSCLC cell lines (SPC-A1, NCI-H358, A549 and PC9) and normal lung 16HBE epithelial cells by qRT-PCR. (**C**) The expression of HOXA-AS2 was measured in cytoplasm and nucleus of A549 cells by qRT-PCR. (**D**) Kaplan–Meier curve analysis revealed that NSCLC patients with high HOXA-AS2 expression had poor survival rate. **P<0.01.

### Knockdown of HOXA-AS2 inhibits proliferation and induces cell apoptosis of NSCLC cells

To investigate the effect of HOXA-AS2 on NSCLC cell biological behavior, we reduced the expression of HOXA-AS2 in A549 cells by transfection with three siRNAs (si-HOXA-AS2#1, #2 and #3). We found that these siRNAs could significantly decrease HOXA-AS2 expression in A549 cells (Figure 2A). si-HOXA-AS2#1 displayed the biggest reduction in A549 cells, thus, it was selected for subsequent experiments, and named as: si-HOXA-AS2. MTS assay revealed that HOXA-AS2 depletion obviously decreased cell proliferation of A549 cells at 48–72 h (Figure 2B). Moreover, flow cytometry assay showed that HOXA-AS2 knockdown significantly induced cell apoptosis of A549 cells (Figure 2C).

**Figure 2:** Knockdown of HOXA-AS2 inhibits proliferation and induces cell apoptosis of NSCLC cells (**A**) The expression of HOXA-AS2 was examined in A549 cells transfected with three siRNAs (si-HOXA-AS2#1, si-HOXA-AS2#2 and si-HOXA-AS2#3) or si-NC by qRT-PCR. (**B**) Cell proliferation was examined in A549 cells transfected with si-HOXA-AS2 or si-NC by MTS assay. (**C**) Cell apoptosis was detected in A549 cells transfected with si-HOXA-AS2 or si-NC by flow cytometry assay. *P<0.05, **P<0.01.

### Knockdown of HOXA-AS2 inhibits cell migration and invasion of NSCLC cells

To explore the effect of HOXD-AS1 on NSCLC metastasis, cell migration and invasion were determined in A549 cells transfected with si-HOXA-AS2. Wound healing assay revealed that knockdown of HOXA-AS2 obviously decreased cell migration abilities of A549 cells (Figure 3A). Consistently, transwell invasion assay demonstrated the invasion capacity of A549 cells was significantly suppressed by HOXA-AS2 depletion (Figure 3B).

**Figure 3:** Knockdown of HOXA-AS2 inhibits cell migration and invasion of NSCLC cells (**A**) Cell migration was detected in A549 cells transfected with si-HOXA-AS2 or si-NC by wound healing assay. (**B**) Cell invasion was detected in A549 cells transfected with si-HOXA-AS2 or si-NC by transwell invasion assay. **P<0.01.

### miR-520a-3p is a target of HOXA-AS2 in NSCLC

Accumulating evidence suggested that lncNRAs exerted biological role in tumor cells via serving as miRNA sponges to negatively regulate miRNAs expression [22,23]. To investigate the possible molecular regulatory mechanism by which HOXA-AS2 exerts oncogenic role in NSCLC, we predicated target miRNA that could interact with HOXA-AS2 by Starbase2.0. We found that HOXA-AS2 contained one conserved target binding site of miR-520a-3p (Figure 4A). To confirm this predication, luciferase reporter assay was conducted in A549 cells co-transfected with the reporter vector (WT/MT HOXA-AS2) and miR-520a-3p mimic or miR-NC. We found that overexpression of miR-520a-3p obviously inhibited luciferase activity of WT-HOXA-AS2 in A549 cells, but not of MT-HOXA-AS2 activity (Figure 4B). RIP experiment demonstrated that HOXA-AS2 and miR-520a-3p were both enriched in Ago2 pellets compared with control IgG in A549 cells (Figure 4C), suggesting that miR-520a-3p could interact with HOXA-AS2 in NSCLC cells. In addition, we found that overexpression of miR-520a-3p significantly decreased HOXA-AS2 expression in A549 cells (Figure 4D). HOXA-AS2 knockdown obviously increased miR-520a-3p expression in A549 cells (Figure 4E). Moreover, we found that miR-520a-3p expression was down-regulated in NSCLC tissues and cell lines (Figure 4F,G), and its expression was negatively correlated with HOXA-AS2 in NSCLC tissues (Figure 4H). These findings implied that miR-520a-3p might be a potential target of HOXA-AS2 in NSCLC.

**Figure 4:** miR-520a-3p is a target of HOXA-AS2 in NSCLC (**A**) Potential binding site and mutant site for miR-520a-3p in HOXA-AS2 is shown. (**B**) Luciferase reporter assay was performed in A549 cells cotransfected with report vector WT-HOXA-AS2 or MT-HOXA-AS2 and miR-520a-3p mimic or miR-NC. (**C**) Cellular lysates from A549 cells were used for RIP with Ago2 antibody, and mouse IgG was used as the control. The expression of HOXA-AS2 and miR-520a-3p was examined using qRT-PCR. (**D**) The expression of HOXA-AS2 was determined in A549 cells transfected with miR-520a-3p mimic or miR-NC by qRT-PCR. (**E**) The expression of miR-520a-3p was determined in A549 cells transfected with si-HOXA-AS2 or si-NC by qRT-PCR. (**F**) The expression of miR-520a-3p in 52 pairs of NSCLC tissues and adjacent normal tissues were examined by qRT-PCR. (**G**) The expression of miR-520a-3p was measured in four NSCLC cell lines (SPC-A1, NCI-H358, A549 and PC9) and normal lung 16HBE epithelial cells by qRT-PCR. (**H**) The correlation of HOXA-AS2 and miR-520a-3p was analyzed using Spearman’s rank correlation analysis. **P<0.01.

### HOXA-AS2 regulates HOXD8 and MAP3K2 by sponging miR-520a-3p

HOXD8 and MAP3K2 have been identified to act as direct targets of miR-520a-3p in NSCLC [24,25]. To investigate whether HOXA-AS2 could affect HOXD8 and MAP3K2 expression by regulating miR-520a-3p, the levels of HOXD8 and MAP3K2 were determined by qRT-PCR and Western blot analysis in A549 cells that were transfected with si-NC, si-HOXA-AS2 with or without miR-520a-3p. As presented in Figure 5A,B, knockdown of HOXA-AS2 led to a prominent reduction in HOXD8 and MAP3K2 expression in A549 cells, while miR-520a-3p partially reversed this trend. In addition, we found that *HOXD8* and *MAP3K2* expression was increased in NSCLC tissues (Figure 5C,D), and their expression were positively correlated with HOXA-AS2 in NSCLC tissues (Figure 5E,F).

**Figure 5:** HOXA-AS2 regulates HOXD8 and MAP3K2 by sponging miR-520a-3p (**A,B**) The expression of HOXD8 and MAP3K2 on mRNA and protein levels were determined in A549 cells transfected with si-NC, si-HOXA-AS2, and si-HOXA-AS2 + miR-520a-3p inhibitor (miR-520a-3p in) by qRT-PCR and Western blot, respectively. (**C,D**) The mRNA expression of *HOXD8* and *MAP3K2* in 52 pairs of NSCLC tissues and adjacent normal tissues were examined by qRT-PCR. (**E,F**) The correlation of HOXA-AS2 and *HOXD8* or *MAP3K2* was analyzed using Spearman’s rank correlation analysis. *P<0.05, **P<0.01.

### Down-regulation of miR-520a-3p partially attenuated the effects of HOXA-AS2 on NSCLC cells

To validate whether HOXA-AS2 affects NSCLC cell proliferation and invasion via regulating miR-520a-3p, A549 cells with si-HOXA-AS2 or si-NC were transfected with the miR-520a-3p inhibitor, then cell proliferation, apoptosis, migration and invasion were determined. Transfection of miR-520a-3p inhibitor could decrease HOXA-AS2 expression in A549 cells transfected with si-HOXA-AS2 (Figure 6A). In addition, down-regulation of miR-520a-3p expression in A549 cells partially reversed the effects of HOXA-AS2 knockdown on cell proliferation, apoptosis, migration and invasion (Figure 6B–E). These data indicate that HOXA-AS2 exerts it biological function in NSCLC by regulating miR-520a-3p.

**Figure 6:** Down-regulation of miR-520a-3p partially attenuated the effects of HOXA-AS2 on NSCLC cells (**A**) The expression of miR-520a-3p were determined in A549 cells transfected with si-NC, si-HOXA-AS2, and si-HOXA-AS2 + miR-520a-3p in by qRT-PCR. (**B**–**E**) Cell proliferation, apoptosis, migration and invasion were determined in A549 cells transfected with si-NC, si-HOXA-AS2, and si-HOXA-AS2 + miR-520a-3p. *P<0.05, **P<0.01.

## Discussion

LncRNAs have access to be involved in NSCLC initiation and development, and serve as tumor suppressor or promoter [9,10]. For example, Zhang et al. [26] showed that PICART1 functioned as a tumor suppressor that suppressed cell proliferation and invasion partly through regulating AKT signaling pathway.Liu et al. reported that LncRNA MAFG-AS1 could promote NSCLC cells growth and metastasis through acting as an miR-339 sponge to regulate MMP15 [27]. Jing et al. [28] demonstrated that CRNDE functioned as an oncogenic lncRNA that promoted NSCLC progression by regulating miR-338-3p. Yuan et al. [29] revealed that LINC01436 acted as a proto-oncogene in NSCLC through functioning as an miR-30a-3p sponge to regulate the its target gene *EPAS1* expression. In the present study, we showed that HOXA-AS2 expression was up-regulated in NSCLC tissues and cell lines. Increased HOXA-AS2 related to clinical features and prognosis of NSCLC patients. In addition, we also found that HOXA-AS2 functioned as a proto-oncogene that contributed to the proliferation and invasion of NSCLC cells by sponging miR-520a-3p. These results suggested that HOXA-AS2 might be a potential target for NSCLC.

Accumulating evidence suggested that lncRNAs exerted tumor suppressive or oncogenic role in cancers usually by regulating serving as miRNA sponges to negatively regulate miRNAs expression [30]. To test molecular mechanism that HOXA-AS2 promoted NSCLC progression, Starbase2.0 was used to predict miRNAs that interact with HOXA-AS2. Among miRNAs, miR-520a-3p was selected based on its biological role in cancer. In NSCLC, miR-520a-3p has been reported to be down-regulated, and was associated with poor prognosis [24,25,31]. Moreover, miR-520a-3p overexpression significantly decreased NSCLC growth and metastasis *in vivo* and *in vitro* [24,25,31], suggesting that miR-520a-3p played tumor suppressive role in NSCLC. Here, luciferase reporter activity and RIP assays confirmed that miR-520a-3p was a downstream target of HOXA-AS2 in NSCLC. A negative correlation with miR-520a-3p and HOXA-AS2 was observed in NSCLC tissues. Furthermore, miR-520a-3p inhibitor partially reversed the effects of HOXA-AS2 knockdown on cell proliferation, apoptosis, migration and invasion of A549 cells. These results suggested that HOXA-AS2 exerts it biological function in NSCLC by regulating miR-520a-3p.

It was well known that lncRNA could indirectly regulate the downstream target of miRNAs by sponging miRNAs [32]. HOXD8 and MAP3K2 were identified to act as two targets of miR-520a-3p in NSCLC [24,25]. Therefore, we investigated whether HOXA-AS2 could affect HOXD8 and MAP3K2 expression by regulating miR-520a-3p. We found that HOXD8 and MAP3K2 expression were up-regualted, and their expression was positively correlated with HOXA-AS2 in NSCLC tissues, respectively. Moreover, knockdown of HOXA-AS2 led to a prominent reduction in HOXD8 and MAP3K2 expression in A549 cells, while miR-520a-3p inhibitor partially reversed this trend. These results implied that HOXA-AS2 could regulate HOXD8 and MAP3K2 expression by sponging miR-520a-3p.

In conclusion, the present study identified HOXA-AS2 as an oncogene lncRNA that contributed to promoting NSCLC progression through the repression of miR-520a-3p. Furthermore, HOXA-AS2 could positively regulate HOXD8 and MAP3K2 expression through regulating miR-520a-3p in NSCLC cells. These findings suggested that HOXA-AS2 might serve as a therapeutic target for NSCLC. Since HOXA-AS2 could target multiple miRNAs or mRNAs, more clinical and experimental studies needed to be performed to further investigate molecular mechanism of HOXA-AS2 in NSCLC.

## Abbreviations

CRNDE: Colorectal Neoplasia Differentially Expressed
FBS: fetal bovine serum
GAPDH: Glyceraldehyde-3-phosphate-dehydrogenase
HOXA: Homeobox A
HOXA-AS2: HOXA cluster antisense RNA 2
HOXD8: Homeobox D8
lncRNA: long noncoding RNA
MAP3K2: Mitogen-activated protein kinase
NSCLC: non-small cell lung cancer
qRT-PCR: quantitative real-time PCR
RIP: RNA immunoprecipitation
si-NC: non-target siRNA control
siRNA: small interfering RNA
